# Important Explorations on Surface Corrosion of the Copper Coins Sourced from the Qing Dynasty

**DOI:** 10.1155/2022/1647217

**Published:** 2022-07-13

**Authors:** Xue Yin, Kang Yang, Honglei Zhang, Bangying Xiong, Mengcheng Duan, Minghao Wang, Yongxing Hao

**Affiliations:** ^1^College of Marxism, Anyang Institute of Technology, Avenue West of Yellow River, Anyang 455000, China; ^2^School of Mechatronic Engineering, Zhengzhou University of Industrial Technology, Zhengzhou 450000, China; ^3^Department of Mechanical Engineering, Anyang Institute of Technology, Avenue West of Yellow River, Anyang 455000, China; ^4^School of Mechanical Engineering, Sichuan University of Science & Engineering, 180# Xueyuan Street, Huixing Road, Zigong 643000, China; ^5^School of Materials Science and Engineering, North China University of Water Resources and Electric Power, Zhengzhou, Henan, China

## Abstract

Surface corrosion is considered to be a main reason for the surface pattern damages of copper coin sourced from the Qing Dynasty. In this study, micromorphology and the structural feature of the copper coins were analyzed to determine their corrosion mechanisms. The results revealed that the etching rates successively reduced with decreasing corrosion thickness, possibly because of unique macrofeatures of the surface pattern. Variable phases, bonding morphologies, and three-/two-dimensional structures of Ql-TB (Qianlong-Tongbao) coins were visibly different at the microscale, which induced disproportional stresses and microscopic cracks, facilitating an unhindered entry of oxide and hydroxyl (OH^−^) ions. These species resulted in the competitive interplay of self-healing and self-degradation mechanisms on the coin surfaces and formed corrosion thickness of ~9.31 *μ*m and a mean corrosion rate of ~2.7%. This study provided an important guideline for preserving microstructures and surface patterns of historical copper coins.

## 1. Introduction

Over the past two decades, extensive research efforts have been devoted toward enhancing the corrosion resistances of various metallic materials. Although significant progress has been acquired in the preservation of copper materials, enhancing their corrosion resistance remains a considerable challenge [1–3]. Under an easy corrosion condition, more than one-third of the copper products are consumed to produce the dissipation [4, 5]. Poor corrosion resistance has limited the applicability of coppers to serve for such corrosive environments like seawater and oxygen-rich humid soil [6, 7]. Therefore, it is imperative to comprehensively investigate the corrosion mechanisms of coppers for preventing surface corrosion of the coins that were produced during the Qing Dynasty.

Coating the copper surface with a protective material is an effective strategy for enhancing the corrosion resistance of copper products [8]. Methods such as phosphate treatment, heavy metal electroplating, mechanical alloying, and ball milling have been widely adopted to fabricate the coatings with satisfactory corrosion resistances [9, 10]. However, large amounts of toxic gases and wastewater, which have adverse effects on the environments, have been generated during these processes. Therefore, numerous studies have focused on developing simple, eco-friendly, and low-cost methods to improve corrosion resistances of copper-based materials. Mousavi and Pitchumani [11] prepared a superhydrophobic surface with multiscaled asperities on a defined copper substrate and achieved a more than fourfold improvement in corrosion resistance, if compared to bare copper. Subsequently, Luo et al. [12] synthesized the new pyridazine derivative, 2-[(6-ethoxy-3-pyridazinyl)thiyl]-*N*,*N*-diethylacetamide (EPD), that served as an efficient corrosion inhibitor for coppers in a sulfuric acid medium and observed maximal inhibition efficiencies of 94.1% at 298 K, 93.2% at 308 K, and 91.3% at 318 K in the presence of 4 mM EPD. The excellent performance was ascribed to the EPD adsorption film formed on a copper surface, in accordance with the Langmuir adsorption isotherm. Dobkowska et al. [13] conducted corrosion tests on copper in an aerated aqueous solution of nitric acid (100 mM). In the case of fine-grained copper, the grain boundaries with high angles and the multihole distributions were established to be the important features that influenced the corrosion rates of copper. Many studies [14–18] have suggested that an optimal grain orientation had a positive effect on copper corrosion, subsequently ensuring crystallographic-orientation-dependent differences in electrochemical corrosion behaviors between coarse-grained material and fine-grained nanocrystalline materials.

As mentioned above, various advanced methods have been developed to prevent the corrosion of copper products, further preventing their surface damage. In recent years, copper coins of the Qing Dynasty have been found to be severely corroded, along with substantial damage to their exquisite structures and microcosmic patterns. This has significantly diminished economic values of these historical coins. But, to the best of our knowledge, corrosion mechanisms of such ancient copper coins have rarely been reported, and understanding these is helpful in developing the protective measures for preventing the corrosion-induced damage of these valuable coins.

In this study, corrosion morphologies, elemental compositions, variable phases, and three-/two-dimensional (3D/2D) microstructures of the copper-prepared coins were comprehensively examined to understand the formation process and growth mechanism of corrosion products. Elemental and phase compositions of the coins were analyzed using energy-dispersive X-ray spectroscopy (EDS) and X-ray diffraction (XRD). Further, surface morphology and 3D/2D microstructures of the corroded coins were evaluated via field emission scanning electron microscopy (FESEM) and the 3D profiler (3DP), respectively. In the end, the formation and growth of the corrosion products were elucidated in depth. Herein, understanding these phenomena was key for protecting the exquisite structural patterns of such coins.

## 2. Sample Source and Main Characterization Techniques

To protect the exquisite structural patterns of the copper coins produced during the Qing Dynasty, Tongbao (TB) coins in the Kangxi (Kx), Jiaqing (Jq), Daoguang (Dg), Tongzhi (Tz), and Qianlong (Ql) periods, which were mainly sourced from private collections (Pr-Cos), were considered as the raw samples, which are shown in Figure 1. The corresponding sample labels were as follows: coin 1: Kx, coins 2–3: Jq, coins 4–5: Dg, coin 6: Tz, and coins 7–11: Ql. In order to obtain the pH values of these coins, the coin surfaces were cleaned for 5 min using ethyl alcohol, and then, a weight ratio of 25.0 : 1.0 for ultrapure water and copper coin was used to soak fifteen coins for 1440 min under room temperature. Subsequently, a well-proportioned mixture of water and coin was carried out for 10 min on an ultrasonic cleaner of model No. KM-12A. Finally, the mixed water was poured into a glass beaker that was placed on the pH instrument of No. EL20. After the calibration, these copper coins were well-detected for four times to acquire the mean pH value.  Table 1 shows the main dimensions (excircle diameter × inner square hole side length) and important characteristics of the coins. As shown in the table, pH levels of the coins ranging from 7.14 to 8.49 confirmed their alkalinity. Unique surface structures of these samples are shown in Figure 1. These photographs in Figure 1 reveal variable dimensions of the examined copper coins. In this study, XRD, FESEM, EDS, and 3DP were adopted as the primary characterization techniques to analyze corrosion products on the coin surfaces. These techniques were appropriate for understanding formation mechanisms and providing insights into the measures to be adopted to conserve such coins.

## 3. Results and Discussions

### 3.1. Corrosion Performances of the Copper Coins

To investigate surface corrosion behaviors of the copper coins shown in Figure 1, the commercial solutions of sodium sesquicarbonate and the hydrogen peroxides with benzotriazole were alternately used to remove the corrosion products of their surfaces to obtain the cleaned coins. Furthermore, 3DP tests were performed to scan surface heights before/after cleaning to determine the height differences, for assessing their etched thickness. Subsequently, the raw (*W*_raw_) and cleaned (*W*_cleaned_) weights of the copper coins were measured carefully; for calculating the weight loss (*W*_loss_), the equation*W*_loss_ = *W*_raw_–*W*_cleaned_was used; furthermore, the corrosion rates (*W*_rate_) of coins could be well calculated as *W*_rate_ = *W*_loss_/*W*_raw_.

Figure 2 presents representative histograms showing the etched thicknesses and their corresponding corrosion rates of the different coins. As shown in these figures, higher etched thickness and corrosion rates were obtained for the Jq copper coin, if compared with the Dg-TB coin, while the Kx coins exhibited excellent corrosion resistance with smaller thicknesses and lower corrosion rates. Maximum etched thickness and the highest corrosion rate could be well observed in the Tz sample; conversely, the lowest corrosion rate was obtained for the Ql coin, indicating the highest corrosion resistance of Ql. Surface etching rates decreased with the reduction of etched thicknesses, which may be due to the close relationship between etching rates and surface structures. An observed variation in corrosion resistance might be due to the unique structures and surface patterns of each coin. Structural patterns of Tz-TB and Ql coins resulted in maximal and minimal etched thicknesses, respectively, of the corroded layers. It caused the Tz and Ql coins to exhibit the lowest and highest corrosion resistances, respectively. For analyzing surface corrosion of the copper coin in greater detail, FESEM was carried out to characterize their surface morphologies.

### 3.2. Surface Analysis of Copper Coins

Unambiguous observations of surface morphologies and microscopic structures were excellent for understanding the copper coin corrosion. Typical FESEM morphologies of the microscopic surfaces of corroded coins are shown in Figure 3. As observed in Figures 3(a)–3(c), small micropores and short microcracks of the Jq coins are clearly visible in Figure 3(b), if compared with those of the Kx coins (Figure 3(a)). As shown in Figure 3(c), fine and long microcracks appeared on the surface of Dg-TB along with large microporous structures that revealed the poor morphology of Dg coin. Furthermore, small micropores and short microcracks facilitated the surface corrosion of the Jq coin, in contrast to dense structures of Kx-TB. Dense microstructures of the latter blocks prevented the corroded particles from entering the coins, thereby hindering surface corrosion. On the other hand, long microcracks and large multiholes significantly aggravated the surface corrosion of the Dg-TB, leading to their poor surface morphologies. Greater numbers of large porous microstructures (~60-250 *μ*m) were observed in Figure 3(d) for Tz-TB than in Figures 3(a)–3(c) for the other samples. This indicated that the Tz coins contained loose corrosion microstructures that caused unexpected corrosion, further leading to the largest etched thickness and highest corrosion rate among the raw samples.

Further, an inset of Figure 3(a) showed an EDS spectrum of a Kx coin, which revealed the main elements comprising the Kx corrosion products. Mass fractions of respective elements in the corrosion products are presented in Table 2; herein, higher mass fractions (wt.%) of Cu, Sn, O, Si, and C presented mass fractions (wt.%) of 22.44, 1.08, 40.64, 10.04, and 19.53, respectively, if compared to small amounts of Al (3.77 wt.%), Ca (2.48 wt.%), and Pd (0.02 wt.%). Similarly, the elemental mass fractions (wt.%) of Jq, Dg, and Tz coins were determined; the results are presented in Table 2. A comparison of the results for Tz-TB with those for the Kx, Jq, and Dg coins revealed that the corrosion products of Tz mainly contained Cu, Sn, O, and Si with different mass fractions, but C was not detected. An absence of C in the Tz coin was not conducive for the formation of the C-containing phase and partially accounted for the poor surface morphologies of the coins with abundant micropores. These pores afforded facile pathways for accelerating the coin surface corrosion, leading to the higher corrosion rate. In the cases of Kx, Jq, and Dg samples, different mass fractions of the main elements resulted in observable variations in the number of phases and their bonding, further forming the observed microdifferences in surface microcracks and microporous structures.

Figure 4 shows the typical micromorphologies of corrosion products of the Ql coins. As can be seen from Figure 4, dense structures (Figure 4(a)), fine cracks (Figure 4(b)), large and long microcracks with small apertures (Figure 4(c)), and porous structures (Figure 4(d)) were ensured in the corrosion surfaces of Ql-TB. Furthermore, numerous microcracks of the coin surface promoted the continuous growth of loose structures, as shown in Figure 4(e). These observed porous and loose microstructures are shown in Figure 4(f), along with many small microholes.

EDS results of the Ql-TB samples indicated that corrosion products were mainly composed of Cu (19.03 wt.%), Sn (11.82 wt.%), O (32.15 wt.%), Si (9.18 wt.%), C (21.65 wt.%), Al (3.53 wt.%), Pb (1.01 wt.%), and Ca (1.63 wt.%). Mass fraction of C in the Ql coin was higher than that in the Kx coin and showed evident differences of C-phase bonding. Moreover, Ql-TB contained a smaller amount of O than the Kx coin. This indicated that smaller amounts of oxides were produced in the former, suggesting less corrosion damage to ensure the excellent corrosion resistance of the Ql coin.

Figure 5(a) exhibits the typical XRD curves of corrosion products on the coin surfaces. Corrosion products of the Tz coin mainly comprised SnO, CuO, Cu_3_Sn, and SiO_2_; no Cu_2_(OH)_2_CO_3_ was detected because of an absence of the C element. Under an alkaline condition, a possible reaction that occurred on its surface was Sn+2OH^−^⟶SnO+H_2_O. This was probable because of the presence of massive hydroxyl ions (OH^−^) in an alkaline atmosphere and resulted in high OH^−^ concentration that induced a chemical reaction of SnO. Meanwhile, the presences of massive oxygen ions resulted in oxygen corrosion via the following pathways: 4Cu+O_2_⟶2Cu_2_O, 2Cu_2_O+O_2_⟶4CuO, 3Cu+Sn⟶Cu_3_Sn, and Si+2O⟶SiO_2_. Constituent elements of the phases identified by XRD were consistent with those identified by an EDS in Table 2, thus confirming the presences of Cu, Sn, O, and Si. It could be concluded that Cu_2_(OH)_2_CO_3_ phases played an important role in determining the thicknesses of the corrosion layer. Thus, an absence of Cu_2_(OH)_2_CO_3_ resulted in higher corrosion rates of the Tz coin than of the Kx, Jq, and Dg coins.

As shown in Figure 5(b), corrosion products of the Ql coins mainly consisted of SnO, CuO, Cu_3_Sn, SiO_2_, and Cu_2_(OH)_2_CO_3_, which were analogous to those of the Kx, Jq, Dg, and Tz samples. Main synthesis of Cu_2_(OH)_2_CO_3_ was represented as follows: 2Cu+O_2_+CO_2_+H_2_O⟶Cu_2_(OH)_2_CO_3_. However, intensities and positions of the diffraction peaks of the Ql corrosion products were ensured to be significantly different, showing that the mass fractions of SnO, SiO_2_, Cu_2_(OH)_2_CO_3_, CuO, and Cu_3_Sn in the Ql coins differed from those in the Kx, Jq, Dg, and Tz samples, according to elemental fractions that are listed in Table 2. This confirmed that different amounts and distributions of the various phases produced the diverse bonding. Hence, unique surface morphologies could be well-observed in the Ql-TB, as can be noted from Figure 4, which resulted in their corrosion rates being lower than those of the other raw coins.

### 3.3. Microstructural Analyses of the Ql Coins

To investigate specific morphologies of the Ql coins, 3D/2D structural analyses for microscopic areas with approximate dimensions of 20 *μ*m × 20 *μ*m were performed.  Figure 6(a) shows a top-view cloud map of the depth simulation of the Ql coin for an area of 20 *μ*m × 20 *μ*m. 3D height distributions and their percentages are shown in Figures 6(b) and 6(c), respectively. As shown in these figures, the data revealed that more than 70% of surface heights were distributed in the range of 1.975-3.951 *μ*m. Main parameters of the heights were as follows: root mean square height (Sq) = 1.126 *μ*m, skewness (Ssk) = −0.628, kurtosis (Sku) = 3.155, maximum peak height (Sp) = 3.539 *μ*m, maximum pit height (Sv) = 4.363 *μ*m, maximum height (Sz) = 7.902 *μ*m, arithmetical mean height (Sa) = 0.877 *μ*m, peak material portion (Smr) = 0.217%, and inverse areal material ratio (Smc) = 1.314 *μ*m. The 2D-linear profile corresponding to the straight line AA of Figure 6(a) is presented in Figure 6(d). According to the statistical results in Figure 6(e), more than 70% of microscopic heights were distributed in the range of 0.417-4.167 *μ*m; among these, the surface heights of 1.249-1.667 *μ*m accounted for ~14%. This result indicated that the smooth surface of the Ql coin was beneficial in preventing oxygen from penetrating the sample, thus improving their corrosion resistance.

To elucidate surface morphologies of the specific regions of Ql coins, their 3D morphologies and structural parameters were analyzed using FESEM.  Figure 7(a) shows the 10 *μ*m × 10 *μ*m area scanned with 251 × 251 testing points at the spacing of 0.04 *μ*m and height of 4.959 *μ*m. Figures 7(b) and 7(c) indicate the top-view cloud map of the depth simulation and the top-view grayscale image of the scanned areas, respectively.  Figure 7(d) depicts the 3D morphology of the scanned area in terms of surface heights, and Figure 7(e) shows the main height distributions. More than 80% of microscopic heights were mainly distributed in this range from 1.24 *μ*m to 2.479 *μ*m. In this case, the percentage of microscopic heights at 2.727-2.851 *μ*m exceeded 8%. 3D heights were analyzed in accordance with the ISO 25178 standard.  Figure 7(f) shows the corresponding parameters and functions of surface heights. Extracted parameters were as follows: Sq: 0.635 *μ*m, Ssk: -0.016, Sku: 2.862, Sp: 2.531 *μ*m, Sv: 2.428 *μ*m, Sz: 4.959 *μ*m, Sa: 0.510 *μ*m, Smr: 0.756%, and Smc: 0.824 *μ*m.

A comparison of Figure 6 with Figure 7 revealed considerable differences in the heights and feature parameters in the corrosion areas, indicating the different microstructures in their respective areas. This may be because the different elements were presented in the varying forms of mass fractions in their microscopic areas, and then, they formed different phases in the corresponding quantities, resulting in the poor bonding of these phases. Such discrepancies caused different morphologies in the corresponding regions, as shown in the FESEM images of Figure 4, further leading to the notable differences in surface corrosion. In other words, different growth rates of the corrosion products led to the formation of different 3D structures on the corrosion surface. Consequently, surface height and feature parameters showed significant differences, according to selected corrosion areas.

## 4. Microcrack Analysis of the Ql Coins

### 4.1. Microscopic Crack Growth of Ql Coins

As mentioned in earlier sections, the growth rates of corrosion products in selected areas of the coins were different and indicated that surface stresses were selectively induced and asymmetrically distributed, resulting in the formation of surface microcracks. Accordingly, studying this phenomenon was an excellent avenue for rationalizing the microcrack formation and its influence on the surface corrosions of Ql coins.  Figure 8 shows the typical FESEM morphologies of etched Ql coins.  Figure 8(a) shows that ~2 *μ*m width cracks formed into the corrosion surface. Further corrosion growth was evidenced due to the harmful formation of long microcracks, as indicated in Figure 8(b). Such punctate corrosion products with small surface microcracks were observed in Figure 8(c).

FESEM morphologies and elemental distributions of the striated corrosion features on the coin surfaces are shown in Figure 9. FESEM morphology of striated corrosion is indicated in Figure 9(a). Distributions of the important phases and overlaid morphologies of the main elements are shown in Figures 9(b) and 9(c), respectively. Microscopic element distributions of oxygen, carbon, and copper on the corrosion surfaces are presented in Figures 9(d)–9(f). The results in Figure 9 revealed that the striated corrosion products were mainly composed of oxygen, carbon, and copper and form two phases, viz., CuO and Cu_2_(OH)_2_CO_3_, as confirmed previously via XRD (Figure 5(b)).

Figure 10 shows the typical FESEM morphologies and elemental distributions of the corrosion products on the Ql coin surface. A subreticulate structure was observed on the corroded surface as indicated in Figure 10(a). Furthermore, Figure 10(b) shows that reticulate corrosion products were distributed on the erosive surfaces. Upon magnifying the reticulate area up to 500 times in the FESEM instrument, small cracks in the reticulate structures became apparent (Figure 10(c)). Upon further magnifying the observed area up to 1000 times, large dendritic cracks were further detected on the corrosion surfaces, as shown in Figure 10(d). Oxygen distributions in the corrosion products are shown in Figure 10(e). As illustrated in Figure 10(f), microcracks formed on the densely organized structures of corrosion products. Based on the previous discussions, it concluded that different corrosion products were formed in different growth areas and produced surface cracks, thereby providing a suitable path for oxygen to enter the Ql coins. The distinct growth rates of the corrosion products accounted for the observed differences in their accumulations and formations of unique structures and FESEM morphologies of the coin surfaces, as indicated in Figures 4 and 10.

### 4.2. Corrosion Mechanisms of the Ql Coins

For analyzing the growth mechanisms of corrosion products on the Ql coin surface, growth models are constructed in Figure 11. Owing to continual contact with oxygen, smooth surfaces of the coins were initially corroded under air, as shown in Figure 11(a). Different corrosion products, SnO, SiO_2_, Cu_2_(OH)_2_CO_3_, CuO, and Cu_3_Sn, formed and grew at different rates in their respective areas, inducing surface stresses in the Ql coins, as shown in Figure 11(b). As illustrated in Figure 11(c), the interior stresses caused an unexpected formation of the surface microcrack. Subsequently, micro-/nanoparticles and oxygen such as carbon and carbonate continually penetrated the microcracks and reacted with the coppers to form the metallic corrosion. The corrosion products grew continuously and then were enriched in the surface cracks, as shown in Figure 11(d). In local areas, different phases of the corrosion products were formed, as shown in Figure 11(e), resulting in different growth rates. Therefore, the corrosion products experienced new stresses in numerous local domains; later, new cracks appeared in the coins at the intersections of old cracks, as shown in Figure 11(f). These newly formed cracks provided favorable conditions for infiltration of oxygen and carbon into the surface cracks of corrosion particles, as illustrated in Figure 11(g), causing subsequent growth of corrosion products. An appreciable growth of corrosion products led to the gradual formation of new microcracks, as indicated in Figure 11(h). These microcracks continued to corrode, expand outwards, and intersect the old cracks to form the striated corrosion products, as shown in Figure 11(i).

Owing to uneven growth of striated corrosion features, new microcracks constantly grew along the striated microstructures and formed dendritic microcracks, as shown in Figure 11(j). As the cracks continued to be corroded, the newly formed cracks intersected the older ones, causing the dendritic structures of microcracks to gradually evolve into subreticulate structures, as shown in Figure 11(k). When corrosion of the Ql coin intensified, subreticulate microstructures of the corrosion products gradually evolved into dense reticulate structures (Figure 11(l)), and new cracks appeared in the reticulate structure as shown in Figure 11(m). With continuous penetration of corrosion particles, the corrosion products grew over the entire coin surface and formed the dense layer in local area, as indicated in Figure 11(n). In the corrosion layers, notable differences of the phase variation, growth rate, and bonding form of corroded surfaces resulted in considerable stress variations. Uneven stress distributions produced new microcracks in the dense corrosion layers, as shown in Figure 11(o). In consequence, the competitive mechanisms operated during the self-healing and self-degradation process of surface microcracks, resulting in the corrosion thickness of ~9.31 *μ*m and mean corrosion rate of ~2.7%.

## 5. Conclusions

In this study, microscopic morphology, structural feature, and corrosion mechanism of the copper coins were examined in detail. Significant insights, which were helpful in preserving the exquisite structures and patterns of copper coins produced during the Qing Dynasty, were acquired. The following four conclusions were drawn:

1. Etching rates of the coins reduced with continuous decreases in the corrosion thickness, likely due to the unique structure of the coin surface, which caused a considerable variation in the corrosion resistance. This in turn caused the Tz and Ql coins to exhibit the lowest and highest corrosion resistances, respectively
2. Variable phase and their bonding in the respective microdomain resulted in the visible differences between the FESEM morphologies and 3D/2D microstructures of the Ql-TB coins, which were not favorable for the uniform stress distributions
3. Inhomogeneous stresses caused formation of microscopic cracks into the Ql coin surface, resulting in loose surface morphologies that facilitated the entry of oxide and hydroxyl ions, thus improving the self-healing capability of the corrosion interface
4. Numerous newly formed microcracks were found in the self-healing surface as a result of poor stress distributions and allowed corrosion products to rapidly grow up to the layer thickness of ~9.31 *μ*m, which corresponded to the mean corrosion rate of ~2.7%

## Figures and Tables

**Figure 1:** Typical copper coins of the Qing Dynasty sourced from private collections (Pr-Co) (1: Kx, 2–3: Jq, 4–5: Dg, 6: Tz, and 7–11: Ql).

**Figure 2:** Typical histograms showing the etched thicknesses (a) and corrosion rates (b) of the copper coins.

**Figure 3:** Typical microscopic surface morphologies of corroded coins observed using FESEM: Kx (a), Jq (b), Dg (c), and Tz (d); an inset in Figure 3(a) showing the EDS profile of corrosion product of the Kx.

**Figure 4:** Representative FESEM morphologies of microscopic surfaces of the Ql coins.

**Figure 5:** Typical XRD curves of the corroded coins sourced from the Qing Dynasty.

**Figure 6:** Typical 3D/2D-morphologies and feature curves of the 20 *μ*m ×20 *μ*m corrosion areas of the Ql coins.

**Figure 7:** Typical 3D morphology and feature parameters of the 10 *μ*m × 10 *μ*m corrosion area of Ql copper coin.

**Figure 8:** Typical FESEM morphologies of the etched Ql coins: microscopic crack (a), crack corrosion (b), and pitting corrosion (c).

**Figure 9:** Typical FESEM results of the striated corrosion products of Ql coins (a) and their element distributions (b–f).

**Figure 10:** Typical FESEM morphologies and element distributions of the etched Ql coin: near-reticulated (a) and reticulated (b) structures, surface microcracks on reticulated structures (c), and dendritic surface cracks (d). Oxygen distribution (e) and microcracks on the dense surface (f).

**Figure 11:** Typical models established for the growth of corrosion layers starting from microcrack generation to formation of striped corrosion features on Ql coin surface.

**Table 1:** Main dimensions (excircle diameter × inner square hole side length) and important characteristics of the coins sourced from the Qing Dynasty.

Series	Source	Coin	pH	Main dimensions	Main characterization techniques
1	Pr-co	Kx	7.44	24.98 mm × 6.31 mm	XRD, FESEM, EDS
2	Pr-co	Jq	7.26	23.04 mm × 6.23 mm	XRD, FESEM, EDS
3	Pr-co	Jq	7.94	23.87 mm × 5.79 mm	XRD, FESEM, EDS
4	Pr-co	Dg	7.41	23.33 mm × 5.02 mm	XRD, FESEM, EDS
5	Pr-co	Dg	7.73	22.39 mm × 5.97 mm	XRD, FESEM, EDS
6	Pr-co	Tz	7.52	21.02 mm × 6.20 mm	XRD, FESEM, EDS
7	Pr-co	Ql	8.49	27.49 mm × 5.88 mm	XRD, FESEM, EDS, 3DP
8	Pr-co	Ql	7.14	25.09 mm × 5.21 mm	XRD, FESEM, EDS, 3DP
9	Pr-co	Ql	7.95	24.13 mm × 5.97 mm	XRD, FESEM, EDS, 3DP
10	Pr-co	Ql	7.84	22.24 mm × 5.96 mm	XRD, FESEM, EDS, 3DP
11	Pr-co	Ql	8.13	22.70 mm × 5.93 mm	XRD, FESEM, EDS, 3DP

**Table 2:** Mass fractions of main elements in the corrosion products on the surfaces of coins produced during the Qing Dynasty.

Copper coins	Elemental mass fractions (wt.%)									
	Cu	Sn	O	Si	C	Al	Pb	Ca	Fe	Pd
Kx-TB	22.44	1.08	40.64	10.04	19.53	3.77	—	2.48	—	0.02
Jq-TB	9.28	2.23	39.19	11.49	21.14	5.05	3.92	1.74	5.97	—
Dg-TB	39.10	2.75	34.09	5.63	18.42	—	—	—	—	0.01
Tz-TB	20.79	5.37	43.71	19.66	—	5.98	4.50	—	—	—
Ql-TB	19.03	11.82	32.15	9.18	21.65	3.53	1.01	1.63	—	—

## Data Availability

The [data type] data used to support the findings of this study are included within the article.
